The article "Effects of Dexmedetomidine on Postoperative Delirium and Expression of IL-1β, IL-6, and TNF-α in Elderly Patients After Hip Fracture Operation" was retracted in 2024. Reason: a breach of policy by an author.

# Effects of Dexmedetomidine on Postoperative Delirium and Expression of IL-1β, IL-6, and TNF-α in Elderly Patients After Hip Fracture Operation

**DOI:** 10.3389/fphar.2020.00678

**Published:** 2020-05-12

**Authors:** Wenchao Zhang, Tianlong Wang, Geng Wang, Minghui Yang, Yan Zhou, Yi Yuan

**Affiliations:** ^1^Department of Anesthesiology, Xuanwu Hospital, Capital Medical University, Beijing, China; ^2^Department of Anesthesiology, Beijing Jishuitan Hospital, Beijing, China; ^3^Department of Orthopaedics & Traumatology, Beijing Jishuitan Hospital, Beijing, China

**Keywords:** dexmedetomidine, elderly patients, hip fracture, pro-inflammatory factor, postoperative delirium

## Abstract

**Objective:**

Postoperative delirium (POD) is a common surgical complication in elderly patients. This study investigated the effects of dexmedetomidine on POD and pro-inflammatory markers in elderly patients with hip fracture.

**Methods:**

This randomized, double-blind, controlled trial enrolled patients ≥65 years of age who underwent an operation for hip fracture at Beijing JiShuiTan Hospital from October 2016 to January 2017. The patients were divided into the DEX group (injected with dexmedetomidine 0.5 µg/kg/h) and the NS group (injected with normal saline). After surgery, the incidence of delirium at postoperative day 1 (T1), 2 (T2), and 3 (T3) was assessed using the Confusion Assessment Method delirium scale. Interleukin (IL)-1β, IL-6, and tumor necrosis factor (TNF)-α blood levels were detected at T0 (before surgery), T1, and T3.

**Results:**

Data from 240 patients were analyzed, with 120/group (intent-to-treat analysis). Dexmedetomidine decreased POD incidence (18.2 vs. 30.6%, P = 0.033). Compared to T0, all three pro-inflammatory markers were higher at T1 and then decreased at T3 (time interaction, all P < 0.001). IL-6 (P < 0.001) levels were lower in the DEX group at T1, and TNF-α (P = 0.003) levels were lower in the DEX group at T1 and T3, but IL-1β levels were similar between the two groups. The rate of adverse events was similar in the two groups.

**Conclusion:**

Dexmedetomidine reduced the incidence of POD in elderly patients on the first day after hip fracture surgery, and reduced IL-6 and TNF-α levels over the first 3 days after surgery.

## Introduction

Postoperative delirium (POD) is an acute confusional state that occurs after an operation under anesthesia, and is characterized by disturbance of consciousness, declined ability to maintain and divert attention, and memory impairment (Numan et al., 2017). Depending on the criteria for diagnosis, the patient population, and the surgical procedure, the incidence of POD ranges 10–70% (Schenning and Deiner, 2015). Alongside the unpleasant experience of POD for the patient, its occurrence also causes other problems. In hospitalized elderly patients, mental disorders such as delirium are associated with longer hospitalization stay, dementia, morbidity, and mortality (Krogseth et al., 2011). As the population age increases, the requirement for surgical procedures increases, especially in the elderly. For instance, the incidence of hip fractures has been increasing in elderly patients, and surgical treatment has to be used in such patients (Robinson et al., 2009). POD is considered to be the most common surgical complication of elderly patients with hip fractures (Bruce et al., 2007; Wang et al., 2015; Yang et al., 2016). In patients undergoing hip fracture surgery, general anesthesia, and subarachnoid (spinal) anesthesia show similar rates of POD (Tzimas et al., 2018).

The occurrence of POD is usually associated with a variety of factors such as advanced aged, preoperative multi-system diseases, medications used in anesthesia, massive blood loss during operation, and pain stimulation (Su et al., 2016). One suggested mechanism for POD is the overexpression of inflammatory responses due to surgical stress leading to the production of proinflammatory cytokines in the brain, resulting in central nervous system inflammatory reaction that affects its function, resulting in POD (Spiegel and Chen, 2012). This theory is supported by the expression of peripheral inflammatory markers in delirium, including C-reactive protein, tumor necrosis factor-alpha (TNF-α), interleukin (IL)-1β, and IL-6 (Gool et al., 2010; Cape et al., 2014; Capri et al., 2014; Cerejeira et al., 2014). Therefore, a possible method to decrease the occurrence of POD could be to decrease the inflammatory response after surgery.

Dexmedetomidine (DEX) is a highly selective α2-receptor agonist that provides sedation, analgesia, and anxiety relief (Keating, 2015). As an α2-adrenergic receptor agonist, DEX can also reduce the systemic inflammatory response and regulate the immune system by inhibiting the central sympathetic nervous system (Tan et al., 2018). A number of studies demonstrated that DEX could reduce the risk of delirium in elderly patients after surgery (Karren et al., 2016; Su et al., 2016; Zeng et al., 2019), but few studies investigated the related changes in pro-inflammatory markers. One study showed that the mechanism of DEX might involve inflammatory responses inhibition, hypoxemia, analgesia, and sleep improvement (Su et al., 2016). Preclinical experimental models showed that DEX could inhibit central inflammatory responses and reduce the production of peripheral serum TNF-α (Xiang et al., 2014). Therefore, DEX might play a role in reducing the incidence of POD in elderly patients undergoing surgery for hip fracture alongside with the levels of pro-inflammatory markers.

This trial aimed to investigate the effects of intraoperative sedation using intravenous DEX on the occurrence of POD in elderly patients operated for a hip fracture. The pro-inflammatory responses alongside the occurrence of POD were explored by detecting expression changes in serum TNF-α, IL-1β, and IL-6 at different time points after surgery.

## Methods

### Patients

This prospective, randomized, double-blind, controlled trial was approved by the Institutional Review Board of Beijing Jishuitan Hospital (Approval No.: 201606-09). The patients signed a written, informed consent form. The clinical trial was registered (ChiCTR-OON-16008691). The study enrolled elderly patients with hip fractures treated at Beijing Jishuitan Hospital from October 2016 to January 2017.

The inclusion criteria were: 1) patients with hip fracture scheduled for operation; 2) 65–90 years of age; and 3) American Society of Anesthesiologists (ASA) physical status scale grade I-III (Sankar et al., 2014).

The exclusion criteria were: 1) patients with a history of psychosis or long-term psychotropic medication use (dementia, schizophrenia), history of chronic analgesic use, or history of alcohol abuse; 2) patients with preoperative mini-mental state examination [MMSE (Li et al., 2016)] score of ≤23, which was assessed at 1 day before surgery (T0); 3) patients who were illiterate; 4) patients with hearing and visual impairments as well as those who had any cerebrovascular accidents such as stroke or transient ischemic attack (TIA) within 3 months; 5) patients with severe infection; or 6) patients with communication barriers who could not complete the cognitive function test.

A computer-generated random number scheme was used to assign the patients into the two groups: the DEX group (n = 110) and the normal saline (NS) group (n = 108).

The patients and researchers (responsible for data recording and analysis, Confusion Assessment Method [CAM (Inouye et al., 1990)] delirium scale assessment, and POD diagnosis) were blinded to the groups, but the anesthesiologists knew about the medication of the patients.

### Anesthetic Management

The patients in both groups underwent proximal femoral nail anti-rotation, cannulated screw fixation, hemiarthroplasty, or total hip arthroplasty. The surgical procedures were performed according to standard procedures. The operations for all patients were performed by the same three surgeons with 5–10 years of surgical experience.

The anesthetic management was the same for both groups of patients except for the administration of DEX. Electrocardiogram (ECG), arterial blood pressure, heart rate (HR), and pulse oxygen saturation (SpO_2_) were monitored after the patients entered the operating room. The patients were in the supine position, and a portable ultrasound unit (WISONIC CLOVER 60VET) with a 4–12 MHz convex array probe was used to identify the femoral artery, femoral nerve, and fascia. The puncture point was 2 cm towards the caudal side from the point at 1/3 the length externally along the line between the anterior superior iliac spine and the pubic tubercle. The in-plane needle approach was applied. After the nerve block needle reached the fascia iliaca compartment, 30 ml of 0.4% ropivacaine were injected. Twenty minutes after the nerve block, the patients were assisted placed in the spinal anesthesia position, with the diseased side on top, and the subarachnoid block was performed in the lateral position. The puncture point was in the L3-4 gap; 12 mg of 0.5 ropivacaine were injected through the subarachnoid space after a successful puncture; otherwise, the puncture was performed between L2-3. All patients underwent subarachnoid block first. If subarachnoid block failed, combined spinal-epidural anesthesia was performed. If lumbar puncture failed (e.g., due to degenerative changes in the spine) or if combined spinal-epidural anesthesia failed, general anesthesia was performed. Etomidate (0.3 mg/kg), sufentanil (0.1 μg/kg), and rocuronium (0.6 mg/kg) were used in general anesthesia. After successful intubation, a ventilator was connected to control breathing. Propofol was continuously infused at 100 mg/h, and sevoflurane was inhaled during the operation to maintain anesthesia. Anesthesia depth was maintained by continuous pumping in 2% sevoflurane and propofol. Dexmedetomidine (0.5 μg/kg/h) was intravenously infused 30 min before the start of anesthesia in the DEX group and was continuously infused at 0.3 μg/kg/h during the operation. The same volume of normal saline was administered for the NS group. The medication was discontinued 30 min before the end of surgery. Propofol was discontinued when the operation was completed. Self-controlled analgesia was performed using patient-controlled intravenous analgesia and sufentanil combined with flurbiprofen ester immediately after the operation.

### Data Collection

Demographics and medical history of the patients were recorded, including sex, age, ASA grade, body mass index (BMI), education level, type of fracture, type of anesthesia, surgical procedure, operation time, and comorbidities.

### Primary Endpoint

The primary endpoint was the incidence of POD, which was assessed at the first postoperative day (T1), the second postoperative day (T2), and the third postoperative day (T3). The patients were first assessed using the Richmond Agitation Sedation Scale (RASS) (Sessler et al., 2002). Those with a RASS >-4 were assessed using the CAM scale to determine the presence of POD. The diagnostic criteria for positive CAM (Inouye et al., 1990) were: (1) acute onset, and fluctuation of the disease condition; (2) distracted attention; (3) thinking disorder; and (4) changes of consciousness. If the patients showed points 1 and 2 and any one of 3 and 4, then CAM was considered positive.

Patients with a positive CAM test at any time point during the follow-up period were screened for delirium within 1 day by a psychiatrist or psychologist based on the Diagnostic and Statistical Manual of Mental Disorders 5 (DSM-5) (Association AP., 2013). Delirium was diagnosed if the following five items were satisfied based on DSM-5: (1) attention deficit disorder; (2) acute onset and repeated changes of symptoms; (3) combined with cognitive impairment; (4) criteria #1 and #3 cannot be explained by existing neurological diseases, and arousal disorder was excluded; and (5) it can be seen from medical history, physical examination, or laboratory tests that it was direct physiological consequences of general physical conditions.

Two trained individuals in our department conducted the assessment of POD, and they were also blind to grouping.

### Secondary Endpoints

#### Biochemical Tests

Five ml of venous blood from the side without infusion were sampled at 9:00 in the morning at T0, T1, and T3, and was centrifuged at 4,000 r/min for 10 min. The serum was separated and stored at −80°C. Before assay, all samples were thawed to room temperature and mixed by gentle swirling or inversion. All samples were assayed on the same day to avoid inter-assay variation. Plasma IL-1β, IL-6, and TNF-α levels were measured by an enzyme-linked immunosorbent assay (ELISA) kit from Bender MedSystems GmbH (Vienna, Austria). This ELISA kit uses the two antibody sandwich ABC-ELISA method. The first antibody was anti-human TNF-α, IL-1β, or IL-6 monoclonal antibody and the second antibody was a monoclonal antibody-containing biotin. Enzyme-labeled streptavidin was bound to the biotin, o-phenylenediamine was added, and the mixture turned yellow. At this time, sulfuric acid was added, and the color became dark. The optical density (OD) value was measured at 492 nm, and the concentrations of TNF-α, IL-1β, and IL-6 were proportional to the OD value. The concentrations of TNF-α, IL-1β, or IL-6 in the specimen were calculated by plotting a standard curve.

The antibodies used in this procedure have no known cross-reactivity with other cytokines. The lowest detectable limits of IL-1β, IL-6, and TNF-α were 1.5 pg/ml, 5 pg/ml, and 1.7 pg/ml, respectively.

#### Numeric Rating Scale (NRS) Scores

Postoperative pain was assessed at T1, T2, and T3 according to a numeric rating scale (NRS), where “0” means no pain at all, and “10” means the worst pain imaginable. Patients with an NRS score of ≥4 after the operation were intravenously injected with 40 mg of parecoxib sodium for analgesia.

### Adverse Events

Invasive arterial blood pressure (systolic [SBP], diastolic [DBP], and mean arterial pressure [MAP]), HR, ECG, and SpO_2_ were routinely monitored during the operation. The number of intraoperative adverse reactions, including hypertension, hypotension, bradycardia, and tachycardia, were recorded. Tachycardia was defined as HR >100 bpm; bradycardia was defined as HR <60 bpm; hypertension was defined as SBP >160 mmHg or 20% of baseline; hypotension was defined as SBP <90 mmHg or 20% of baseline. Patients with bradycardia were administered with 0.1–0.3 mg of atropine, and patients with hypotension were intravenously injected with 4 µg of norepinephrine or intravenously infused at 200 µg/h.

### Statistical Analysis

The incidence of POD in a comparable patient population of a previous study was 28% (Robinson et al., 2009). Therefore, we assumed that the incidence of delirium would be reduced by one third in the DEX group in this trial. With significance set at 0.05 and power set at 80%, the sample size required to detect differences was 196, calculated with the Pass 11.0 software (NCSS, LLC. Kaysville, Utah, USA). Taking into account a lost-to-follow-up rate of about 6%, we planned to enroll 208 patients.

Continuous data with a normal distribution were presented as means ± standard deviation (SD) and analyzed using the independent t-test; those with a non-normal distribution were presented as medians (interquartile range) and analyzed by the Mann-Whitney U-test. Categorical variables were presented as frequencies and percentages and analyzed with the chi-square test or Fisher’s exact test. Repeated measurement analysis of variance was used to analyze the levels of pro-inflammatory markers. Statistical analyses were done on SPSS 22.0 Windows (IBM Corp., Armonk, NY, USA) with two-tailed tests wherever appropriate and P < 0.05 being considered statistically significant.

### Quality Control

The exactness of the data was monitored by the Quality Control division of the Clinical Research Ethics Committee of Beijing Jishuitan Hospital.

## Results

### Patient Inclusion

The intent-to-treat (ITT) analyses are presented here, and the per-protocol (PP) analyses are presented as **Supplementary Material**. A total of 402 patients were assessed for eligibility; 162 patients were excluded based on the inclusion criteria or because they declined participation. The remaining 240 patients were randomly assigned to the DEX or NS group (120/group) (**Figure 1**).

**Figure 1:** Flowchart of study inclusion, randomization, and follow-up.

### Demographics and Medical History

The patients in the DEX group were 78.1 ± 6.4 years of age and 30.8% were male. The patients in the NS group were 79.0 ± 6.8 years of age and 31.7% were male. There were no significant differences between the two groups in demographics, including age, sex, BMI, total education years, ASA grade, comorbidities, type of fracture, anesthesia, surgical procedure, operation time, and time interval between fracture and the operation (all P > 0.05) (**Table 1** and **Supplementary Table 1**). Parecoxib did not have to be used in any patient.

**Table 1:** Demographics and medical history in the ITT analysis.

Characteristics	NS group (N = 120)	DEX group (N = 120)	P
**Age (years)**	79.0 ± 6.8	78.1 ± 6.4`	0.674
**Sex (male)**	38 (31.7%)	37 (30.8%)	0.889
**BMI (kg/m^2^**)	24.2 ± 3.0	23.8 ± 2.5	0.213
**Total education years**			0.355
<5	80 (66.7%)	70 (58.3%)	
5–8	25 (20.8%)	34 (28.3%)	
>8	15 (12.5%)	16 (13.3%)	
**ASA grade**			0.873
I	9 (7.5%)	7 (5.8%)	
II	77 (64.2%)	78 (65.0%)	
III	34 (28.3%)	35 (29.2%)	
**Operation time (min)**	60.0 (40.0–70.0)	60.0 (40.0–70.0)	0.761
**Comorbidities**			
Hypertension	69 (57.5%)	68 (56.7%)	0.896
Diabetes	24 (20.0%)	35 (29.2%)	0.099
Heart failure	9 (7.5%)	9 (7.5%)	1.000
Lung infection	1 (0.8%)	5 (4.2%)	0.215
Chronic bronchitis	6 (5.0%)	7 (5.8%)	0.776
Atrial fibrillation	3 (2.5%)	7 (5.8%)	0.196
Arrhythmia	5 (4.2%)	10 (8.3%)	0.182
**Anesthesia**			0.216
Subarachnoid block	98 (81.7%)	103 (85.8%)	
Combined spinal-epidural anesthesia	17 (14.2%)	16 (13.3%)	
General anesthesia	5 (4.2%)	1 (0.8%)	
**Type of fracture**			0.414
Femoral neck fractures	59 (49.2%)	49 (40.8%)	
Intertrochanteric fracture	59 (49.2%)	68 (56.7%)	
Subtrochanteric fractures	2 (1.7%)	3 (2.5%)	
**Surgical procedure**			0.460
PFNA	61 (50.8%)	54 (45.0%)	
Cannulated screw fixation	32 (26.7%)	28 (23.3%)	
Hemi-arthroplasty	15 (12.5%)	22 (18.3%)	
THA	12 (10.0%)	16 (13.3%)	
**Time interval between fracture and the operation (days)**	2.7 ± 1.2	2.5 ± 1.4	0.184

ITT, intent-to-treat; NS, normal saline; DEX, dexmedetomidine; BMI, body mass index; ASA, American Society of Anesthesiologists physical status scale grade; PFNA, proximal femoral nail anti-rotation; THA, total hip arthroplasty.

### Incidence of POD and NRS Scores

There was a lower incidence of POD at T1 in the DEX group compared with the NS group (13.3 vs. 25.8%, P = 0.015) and in total POD in the DEX group compared with the NS group (16.7 vs. 30.0%, P = 0.015). The POD incidence decreased in both groups with time and was similar at T2 (3.3 vs. 5.0%, P = 0.518) and T3 (1.7 vs. 2.5%, P > 0.99). The NRS scores were similar between the two groups at T1, T2, and T3 (all P > 0.05) (**Table 2** and **Supplementary Table 2**).

**Table 2:** Incidence of POD and NRS scores after surgery in the ITT analysis.

	NS group (N = 120)	DEX group (N = 120)	P
**POD**			
T1	31 (25.8%)	16 (13.3%)	0.015
T2	6 (5.0%)	4 (3.3%)	0.518
T3	3 (2.5%)	2 (1.7%)	1.000
Total	36 (30.0%)	20 (16.7%)	0.015
**NRS**			
T1	2.0 (2.0–3.0)	2.0 (2.0–3.0)	0.239
T2	1.0 (1.0–1.2)	1.0 (1.0–1.0)	0.356
T3	1.0 (1.0–1.0)	1.0 (1.0–1.0)	0.418

ITT, intent-to-treat; POD, postoperative delirium; NS, normal saline; DEX, dexmedetomidine; NRS, numeric rating scale; T1, 1 day after surgery; T2, 2 days after surgery; T3, 3 days after surgery.

### Pro-Inflammatory Markers

The changes in pro-inflammatory markers in the two groups are shown in **Figure 2** and **Table 3**. There were no differences between groups at T0 in all three markers (all P > 0.05). The IL-1β serum concentration changes were similar in both groups and remained above the T0 level at T1 and T3, while both groups showed a significant difference with time (P < 0.001). The serum IL-6 concentration was increased at T1 and T3 compared with T0. The DEX group showed lower serum IL-6 concentrations than the NS group at T1 but similar at T3 (P < 0.001). In both groups, serum TNF-α concentration increased at T1 and T3, but the DEX group showed lower TNF-α concentrations than the NS group at T1 and T3 (P = 0.003) (**Table 3** and **Supplementary Table 3**).

**Figure 2:** Changes in interleukin (IL)-1 **(A)**, IL-6 **(B)**, and tumor necrosis factor (TNF)-α **(C)** levels over time.

**Table 3:** Levels of IL-1β, IL-6, and TNF-α in the ITT analysis.

	NS group (N = 120)	DEX group (N = 120)	F(group)/P-value	F(time)/P-value	F(group*time)/P-value
**IL-1β**					
T0	5.19 ± 0.64	5.10 ± 0.68	*F* = 0.084	*F* = 1330.336	*F* = 0.666
T1	10.88 ± 1.43^a^	11.05 ± 1.79^a^	*P* = 0.773	*P* < 0.001	*P* = 0.492
T3	7.99 ± 1.20^a^ ^b^	7.99 ± 1.25^a^ ^b^			
**IL-6**					
T0	22.94 ± 5.11	23.71 ± 5.58	*F* = 242.373	*F* = 2197.895	*F* = 33.220
T1	105.15 ± 15.35^a^	89.04 ± 10.37^#^^a^	*P* < 0.001	*P* < 0.001	*P* < 0.001
T3	63.26 ± 20.93^a^ ^b^	61.36 ± 15.61^a^ ^b^			
**TNF-α**					
T0	4.35 ± 0.69	4.40 ± 0.74	*F* = 10.666	*F* = 88.084	*F* = 6.478
T1	5.37 ± 0.81^a^	4.93 ± 0.87^#^^a^	*P* = 0.001	*P* < 0.001	*P* = 0.002
T3	4.47 ± 0.85^a^ ^b^	4.19 ± 0.88^#^^a^ ^b^			

ITT, intent-to-treat; NS, normal saline; DEX, dexmedetomidine; T0, 1 day before surgery; T1, 1 day after surgery; T3, 3 days after surgery; IL, interleukin; TNF, tumor necrosis factor.

^#^P < 0.05 vs. the NS group.

a P < 0.05 vs. T0.

b P < 0.05 vs. T1.

### Adverse Events

In total, 102 adverse events were recorded: 44 in the NS group and 58 in the DEX group. These included tachycardia, bradycardia, hypertension, and hypotension. The rates were similar in the two groups (all P > 0.05) (**Table 4** and **Supplementary Table 4**).

**Table 4:** Intraoperative adverse events in the ITT analysis.

	NS group (N = 120)	DEX group (N = 120)	P-value
Tachycardia	10 (8.3%)	9 (7.5%)	0.811
Bradycardia	18 (15.0%)	20 (16.7%)	0.724
Hypertension	16 (13.3%)	22 (18.3%)	0.289
Hypotension	8 (6.7%)	10 (8.3%)	0.624

ITT, intent-to-treat; NS, normal saline; DEX, dexmedetomidine.

## Discussion

The aim of this trial was to investigate the effects of DEX on POD and the levels of pro-inflammatory markers in elderly patients undergoing surgery for hip fractures. Data from 218 patients were analyzed, with 110 patients in the DEX group and 108 in the NS group. The POD incidence was 18.2% with DEX, compared with 30.6% in the NS group. IL-1β, IL-6, and TNF-α serum levels all increased at T1 and then decreased by T3. The IL-6 and TNF-α levels in the DEX group were lower than in the NS group, but IL-1β levels were similar. The rate of adverse events was similar. These results show that DEX reduced the incidence of POD in elderly patients with a hip fracture at 1 day after surgery and reduced the short-term increases in IL-6 and TNF-α concentrations post-surgery. There were no differences in conclusions between the ITT and APP analyses.

Our results suggest that intravenous administration of DEX during surgery significantly reduces the incidence of POD in elderly hip fracture. This result agrees with numerous other studies that also showed reduced rates of POD in elderly surgical patients (Karren et al., 2016; Su et al., 2016; Zeng et al., 2019). By monitoring the serum pro-inflammatory cytokines IL-1β, IL-6, and TNF-α at different time points, we also aimed to investigate the expression of postoperative pro-inflammatory cytokines with DEX administration and the occurrence of POD. Few studies undertook the investigation of cytokines during DEX treatment to prevent POD. A study of 354 patients >65 years of age undergoing laparoscopic major non-cardiac surgery under general anesthesia found that POD was reduced and IL-6 levels were significantly lower at 1 and 24 h when DEX was administered as a bolus before surgery and by infusion from induction of anesthesia to the end of surgery (Lee et al., 2018). For 40 patients undergoing robot-assisted laparoscopic radical cystectomy and ileal conduit diversion, the levels of TNF-α, NSE, and IL-6 in the DEX group were significantly lower than in the control group at 1 and 5 days after the operation (Ding et al., 2015). In young patients, the combined usage of DEX and sufentanil was investigated to treat POD after general anesthesia (Liu et al., 2018). The results showed that the levels of IL-6 and TNF-α were lower at 1 and 8 h after surgery. When the results of these studies and our results are taken together, there is a suggestion that there might be a relationship between pro-inflammatory markers and POD. In our study, on the 1st day after surgery, the levels of IL-1β, IL-6, and TNF-α were relatively high, and the incidence of POD was also relatively high (26.85 and 14.55%). On the 3rd day, the levels of IL-1β, IL-6, and TNF-α were lower, and the incidence of POD dropped to 2.78 and 1.82%. Nevertheless, further studies are needed to investigate whether there is a direct correlation between POD and cytokine levels.

The pathological mechanism of POD is still unclear, and it may be caused by multiple factors. Inflammatory responses and neuroinflammation seem to be the main cause. Therefore, DEX, as an α-receptor agonist, can prevent the occurrence of POD. Elderly patients with hip fractures often have agitation during surgery due to trauma and discomfort caused by their positioning, especially patients receiving intramedullary needle fixation. The sedative effect of DEX can reduce the patient’s agitation during the operation. There is some concern that the application of DEX has many potential side effects, including hypotension, bradycardia, and inhibition of the cardiac conduction system. For elderly patients with hip fractures, it has been suggested that DEX should be administered at the lowest possible doses for the shortest possible time. In our experiment, the initial dose was 30 µg for elderly patients with hip fracture, the infusing dose was 0.2 µg/kg/h, and medication was discontinued 10 min before the end of the operation. In respect to safety, our data revealed that DEX-induced bradycardia and hypotension were not significantly increased, possibly because of the very low doses that were used.

There were several limitations to this study. First, this was a single-center study, and there might be selection and treatment biases. Indeed, all patients were treated by the same team and local practices and personal experience could have influenced the management of the patients, limiting the generalizability of the results. The hospital was a tertiary center and the patients had a good economic condition. In addition, the selection criteria restricted the eligible patients and the results might not be applicable for all elderly patients with hip fracture. Second, the pro-inflammatory indicators were measured at only three time points, and blood specimens were not collected immediately before anesthesia and immediately after anesthesia. Third, the follow-up time was short (only 3 days), which was mainly because hospitalization was short, and blood samples could not be obtained effectively after discharge. Fourth, even if the peripheral levels of pro-inflammatory markers reflect the inflammatory state of the central nervous system, future studies should measure markers that are specific for brain inflammation. Finally, the NRS and blood markers for the patients who were lost to follow-up were not available, and the mean/median method was used for the imputation of the missing data.

## Conclusion

DEX reduced the incidence of POD in elderly patients at 1 day after surgery for hip fractures. DEX also significantly alleviated the increase in short-term IL-6 and TNF-α levels. DEX may benefit patients by reducing the incidence of early POD and offering a better short-term recovery for elderly patients undergoing hip arthroplasty.

## Data Availability Statement

The datasets generated for this study are available on request to the corresponding author.

## Ethics Statement

The studies involving human participants were reviewed and approved by the Institutional Review Board of the Beijing Jishuitan Hospital. The patients/participants provided their written informed consent to participate in this study.

## Author Contributions

Each author has made an important scientific contribution to the study and is thoroughly familiar with the primary data. All authors listed have read the complete manuscript and have approved submission of the paper.

## Funding

This study was supported by Beijing Jishuitan Hospital Nova Program [no. xkxx201619], Capital’s Funds for Health Improvement and Research [2018-1-2071], and Beijing Municipal Administration of Hospitals Clinical Medicine Development of Special Funding Support [ZYLX201813].

## Conflict of Interest

The authors declare that the research was conducted in the absence of any commercial or financial relationships that could be construed as a potential conflict of interest.
